RETRACTED

# Application of Artificial Neural Network Algorithm in Facial Biological Image Information Scanning and Recognition

**DOI:** 10.1155/2022/1142682

**Published:** 2022-09-09

**Authors:** Zexin Zhang, Ruimin Hu, Wenyi Hu

**Affiliations:** ^1^National Engineering Research Center for Multimedia Software, Wuhan, Hubei 430072, China; ^2^School of Computer Science, Wuhan University, Wuhan, Hubei 430072, China

## Abstract

In order to solve the problem that the accuracy of face recognition is not good due to the influence of jitter and environmental factors in the mobile shooting environment, this paper proposes the application of an artificial neural network algorithm in the information scanning and recognition of face biological images. The spatial neighborhood information is integrated into the amplitude detection of multipose face images, and the dynamic corner features of multipose face images are extracted. The structural texture information of multipose face images is compared to a global moving RGB three-dimensional bit plane random field, and the multipose face images are detected and fused. At different scales, appropriate feature registration functions are selected to describe the feature points of multipose face images. The parallax analysis of target pixels and key feature detection of multipose face images are carried out. Image stabilization and automatic recognition are realized by combining artificial neural network learning and feature registration methods. The experimental results show that the experiment is designed with MATLAB, the frame frequency of dynamic face image acquisition is 1200 kHz, the number of collected samples of the multipose face image is 2000, the training sample set is 200, the noise coefficient = 0.24, the number of multipose face image blocks is 120, and the structural similarity is 0.12. It is found that the output signal-to-noise ratio of multipose face image recognition using the method in this paper is high. *Conclusion*. This method has good performance in feature point registration and high recognition accuracy for multipose face image recognition.

## 1. Introduction

Since the end of the last century, the production of digital media has gradually increased. From 2011 to 2012, machine learning algorithms based on inductive statistics were widely used by integrating training materials and improving image processing equations. Deep neural networks are far more efficient than power tools in terms of product cognition, storage, and other locations, and can achieve levels of impact utilization. Then facial recognition technology is passed on to humans. In addition, the demand for business and investment has led to a rapid increase in knowledge about the value cycle of in-depth research, production, education, and research. Biometrics are tools for machine learning algorithms for the study and identification of specific biological species, especially humans [1]. This applies not only to the use of physical features of the human body, such as fingers, palms, face, and iris but also to the use of walking, behavioral, and other techniques of evaluation behavioral factors. In recent years, a wide range of terms have been divided into behavioral descriptions, such as facial expressions based on soft biometrics. In fact, the knowledge of biometrics was the first introduction to machine learning and has been a hotbed of computer vision for the last decade. Compared to other things, the human face has a very rich material. Personal identification information usually depends on the shape of the face. Compared to behavioral and voice knowledge, it is more accurate, faster, and can meet most security needs. In addition, facial recognition is a passive noncontact device that works well because it has little effect on normal operations and does not require victim intervention. However, negative identification marks, such as palm prints and fingerprints, are often opposed [2]. The wide range of cameras and the widespread use of their mobile devices can eliminate the need to install special equipment, saving on purchase costs and reducing support. Although face recognition is easy and fast, it can have many participants. For example, passive recognition is often difficult to capture without focus, like a blurry, motionless swing, and the lighting and text often change. It is worth noting that as modern lifestyles improve, hair color, and hairstyles often change, especially for women, making the process of recognition difficult. In addition to taking a single photo, the popularity of filming equipment and reduced storage costs, as well as the ability to use multiple films for facial analysis. In addition, setting up a face recognition system using one-person photos and videos provides more information and brings more class changes. This makes it difficult to aggregate data [3].

RETRACTED

## 2. Literature Review

In the traditional face recognition methods, the features of face images usually need to be discriminated against and acquired artificially. As an artificial intelligence technology, deep learning abandons manual and repeated feature acquisition operations and focuses on machine learning of features. Deep learning of features is to use hierarchical networks to obtain feature information and build a learning framework by combining multiple core algorithms. Algorithms include rotary neural networks, automatic encoders, limited Boltzmann machines (RBMs), deep communication networks (DBNs), and multilayer input repeater neural networks (RNNs). For many real-life issues, such as images, text, and sound, we can define them in different ways.

Benouis developed the Swets method into the Figenface method. At present, there are many widely used methods in face recognition, of which a large number of researchers use this algorithm. Many popular methods are developed on this [4]. Kadum proposed a convolutional neural network, which is characterized by the convolution layer involved in the depth model. The structure of the convolutional neural network includes the convolutional layer, the downward sampling layer, and the entire connection layer. Although the number of each layer can be adjusted according to the actual situation, the hidden procedure must be at least 5. The earliest and best processing for small-scale image processing at home and abroad is obtained by convolutional neural network analysis [5]. Ergin put forward the Hopfield neural network model, which means laying a good theoretical foundation for the study of artificial neural networks [6]. Until Sun put forward a convolution neural network model with more dimensions after unremitting exploration, which better solved the world-famous Imagenet problem and achieved good results. With the improvement of the CNN model, a convolutional neural network has successfully stood firm in the field of image processing [7]. Gunawan entered the field of face recognition to explore. As early as the 1970s, extracting the set features of side faces became a typical core task of pattern recognition. However, limited by the conditions at that time, the number of features obtained by image processing is small. Even through automatic feature extraction, it is difficult to ensure the accuracy of the extraction [8]. Cuevas focused on image segmentation and image feature extraction. At the same time, they used more traditional data statistical techniques, such as the Karhunen–Loeve transform, to conduct in-depth research on neural network classifiers [9].

This article introduces a multidimensional recognition algorithm based on neural network education. As can be seen from Figure 1, the surrounding spatial information was combined to detect the multiface image amplitude, the angular properties of the multiface image were isolated, and the appropriate feature recording function was selected to describe the multi-face content. Images of various scales, objective pixel parallax analysis, and multidimensional image detection were found to be important. Image stabilization and automatic recognition are achieved through a combination of neural network training and special recording capabilities. From the point of view of simulation, the advantage of this model is that it improves the ability to detect real faces.

RETRACTED

## 3. Research Methods

### 3.1. Multipose Face Image Acquisition and Feature Preprocessing

#### 3.1.1. Face Image Imaging Processing

In order to realize the multipose face image recognition, combined with the image imaging technology to detect and extract the biological attributes of the image, firstly, the laser 3D scanning method is used to image the multipose face image. Assuming that the texture information and pixel feature components of the collected multipose face image are recorded as $v_{m}=\left({\bar{R}}_{m},{\bar{G}}_{m},{\bar{B}}_{m}\right)$ and ${aux}_{m}\left({\hat{I}}_{m},{\tilde{I}}_{m},f_{m},\lambda_{m},{df}_{m},{dl}_{m}\right)$ respectively, and the gray pixel values of the multipose face image are recorded as Ψ_11_, Ψ_12_, Ψ_13_, Ψ_14_ , Ψ_15_, the fuzzy feature recognition method is used to decompose the edge features of the multipose face image, and the edge pixel values are obtained as *η*={*η*_*ij*_ : (*i*, *j*) ∈ *S*, *η*_*ij*_ ∈ *S*}. The points to be detected for feature extraction of multipose face images can be divided into four categories: isolated points, endpoints, continuous points, and bifurcation points.

The pixel intensity of the exposure area block of the face image is as follows:

(1) $$\begin{array}{c} g\left(t\right)=\sqrt{s}f\left(s\left[t-\tau \right]\right)\text{,} \end{array}$$

*f*(*t*) is the high frequency part of the face image; *s*=(*c* − *v*)/(*c*+*v*) represents the edge scale factor of multipose face image; and $\sqrt{s}$ is the normalization factor.

The manual annotation method is used for the scale decomposition of the face image, and the wavelet scale decomposition method is used for image denoising. The wavelet function is as follows:

(2) $$\begin{array}{c} W_{\psi }y\left(a,b\right)=\langle y,\psi_{a,b}\rangle =\overset{+\infty }{\underset{-\infty }{\int }}y\left(t\right)\frac{1}{\sqrt{\left|a\right|}}\psi^{*}\left(\frac{t-b}{a}\right)dt\text{.} \end{array}$$

Using local binary fitting, the geometric dispersion of the face is obtained as follows:

(3) $$\begin{array}{c} \psi_{a,b}\left(t\right)=\left[U\left(a,b\right)\psi \left(t\right)\right]=\frac{1}{\sqrt{\left|a\right|}}\psi \left(\frac{t-b}{a}\right), \end{array}$$

*U*(*a*, *b*) is the unitary transformation function of multipose feature components of the face image.

The block matching method is used for image information fusion. Let *a*=1/*s*, *b*=*τ*, and rewrite equation (3) as follows:

(4) $$\begin{array}{c} f_{s,\tau }\left(t\right)=\left[U\left(1/,\tau \right)f\left(t\right)\right]=\sqrt{\left|s\right|f\left(s\left(t-\tau \right)\right)}\text{,} \end{array}$$

Combined with the template matching method, the edge contour of the biometric feature distribution of the face is obtained as follows:

(5) $$\begin{array}{c} u\left(t\right)=\frac{1}{\sqrt{T}}rect\;\frac{t}{T}\exp\;\left\{-j\left[2\pi K\;\ln\;\left(1-\frac{t}{t_{0}}\right)\right]\right\}, \end{array}$$

where rect(*t*) = 1, |*t*| ≤ 1/2.

RETRACTED

Carry out vector quantization feature decomposition on the collected original multipose face image, and combine the gray manifold segmentation technology to extract the edge contour feature of the multipose face image, so as to improve the ability of face feature extraction [10].

#### 3.1.2. Edge Contour Detection of Multipose Face Images

The spatial neighborhood information is integrated into the amplitude detection of multipose face images, the dynamic corner features of multipose face images are extracted, and the image histogram is constructed. The histogram distribution function is obtained as follows:

(6) $$\begin{array}{c} \theta \left(t\right)=2\pi \int_{-T/2}^{t/a}\left(\frac{K}{t_{0}-t}\right)dt=-2\pi K\;\ln\;\left(1-\frac{t}{at_{0}}\right)+\theta_{0}\text{,} \end{array}$$

where *θ*_0_=−2*πK*ln(1+*T*/2*t*_0_), 

The gray histogram segmentation method is used to segment the multipose face image to improve the feature extraction ability of the multipose face image. The feature points of the face are located according to the edge contour information of the image. The output of face feature extraction is as follows (7):

(7) $$\begin{array}{c} \left[\begin{array}{c} x^{\prime }\\ y^{\prime }\\ 1 \end{array}\right]=\left[\begin{array}{ccc} 1 & 0 & 0\\ 0 & \frac{\delta^{*}\;\sin\;\alpha }{\sin\;\left(\alpha -\theta \right)} & \frac{n}{2\;\cos\;\alpha }-\frac{\delta^{*}{\text{ nose}}^{*}\;\sin\;\alpha }{\sin\;\left(\alpha -\theta \right)}\\ 0 & 0 & 1 \end{array}\right]\left[\begin{array}{c} x\\ y\\ 1 \end{array}\right]\text{.} \end{array}$$

In combination with the biological feature invariance of the face, the noise separation output binary image of the face is obtained, and the result is as follows (8):

(8) $$\begin{array}{c} M=\left[\begin{array}{cc} u_{11} & u_{12}\\ u_{21} & u_{22} \end{array}\right]\\ =u\left(x,y,\sigma_{I},\sigma_{D}\right)\\ =\sigma_{D}^{2}G\left(\sigma_{I}\right)*\left[\begin{array}{cc} L_{x}^{2}\left(x,y,\sigma_{D}\right) & L_{x}L_{y}\left(x,y,\sigma_{D}\right)\\ L_{x}L_{y}\left(x,y,\sigma_{D}\right) & L_{y}^{2}\left(x,y,\sigma_{D}\right) \end{array}\right], \end{array}$$

where *G*(*σ*_*I*_) represents the pixel intensity of the exposure area block of the multipose face image; For the edge pixel (*x*, *y*), *σ*_*I*_ is used to represent the edge wheel integral scale of the multipose face image, *σ*_D_ is the differential scale, and *x*, *y* is the binary pixel of the original image sequence; *L*(*x*, *y*, *σ*_*D*_) represents the information entropy in the image sequence, *L*_*x*_(*x*, *y*, *σ*_D_) and *L*_*y*_(*x*, *y*, *σ*_D_) represent the weight fusion results of the multipose face image in the horizontal translation *x* direction and the vertical translation *y* direction respectively, *L*_*xx*_(*x*, *y*, *σ*_D_) and *L*_*yy*_(*x*, *y*, *σ*_D_) are the cross-correlation feature quantities of the corner distribution of the face [11].

RETRACTED

According to the above analysis, the dynamic corner features of multipose face images are extracted, and the geometric difference eigenvalues of faces are calculated for face feature analysis and classification recognition.

### 3.2. Optimization of Face Feature Extraction and Recognition Algorithm

#### 3.2.1. Feature Extraction of Face Image

On the basis of face image imaging processing and edge contour detection, the recognition algorithm of the face image is optimized [12, 13]. This paper presents a multipose face image recognition algorithm based on artificial neural network learning. The multipose face image structure texture information is compared to a global moving RGB three-dimensional bit plane random field, a feature extraction template is determined, and the feature points that can best reflect the face features are extracted from the image. The RGB feature decomposition formula of the multipose face image is obtained as follows (9):

(9) $$\begin{array}{c} J_{1}\left(W_{i}\right)=\overset{t}{\underset{r=1}{\sum }}\overset{k_{1}}{\underset{p=1}{\sum }}{\left\|W_{i}^{T}x_{iv}-W_{i}^{T}x_{ip}^{\prime }\right\|}^{2}A_{ip}=\\ \overset{t}{\underset{r=1}{\sum }}\overset{k_{1}}{\underset{p=1}{\sum }}tr\;\left(W_{i}^{T}x_{ir}-W_{i}^{T}x_{irp}^{\prime }\right){\left(W_{i}^{T}x_{ir}-W_{i}^{T}x_{irp}^{\prime }\right)}^{T}A_{irp}=\\ \left.\left.\overset{t}{\underset{r=1}{\sum }}\;\overset{k_{1}}{\underset{p=1}{\sum }}\;tr\;\left(W_{i}^{T}\left[\left[x_{ir}\right)\right)-x_{ip}^{\prime }\right){\left(x_{ir}-x_{ipp}^{\prime }\right)}^{T}A_{irp}\right]W_{i}\right)=\\ tr\;\left(W_{i}^{T}\left[\overset{t}{\underset{r=1}{\sum }}\overset{k_{1}}{\underset{p=1}{\sum }}\left(x_{ir}-x_{ipp}^{\prime }\right){\left(x_{ir}-x_{ipp}^{\prime }\right)}^{T}A_{irp}\right]W_{i}\right)=\\ tr\;\left(W_{i}^{T}H_{1}W_{i}\right), \end{array}$$

where *H*_1_=∑_*r*=1_^*t*^∑_*p*=1_^*k*_1_^(*x*_*ir*_ − *x*_*irp*_′)(*x*_*ir*_ − *x*_*irp*_′)^T^*A*_*irp*_ represents the edge feature value of the input multipose face image; *A*_*irp*_ represents the face feature value in the Delaunay triangle region; TR represents the pixel trace of multipose face image feature tracking recognition; *W*_*i*_^T^ represents the relevant characteristic value of the nearest neighbor region [14].

RETRACTED

The information restoration is performed according to the local features of the multipose face image, and the Potts prior parameter *β*_*i*_ of the multipose face image feature detection is obtained as follows (10):

(10) $$\begin{array}{c} \beta_{i}=\exp\;\left\{-\frac{{\left|x_{i}-x_{j}\right|}^{2}}{2\sigma^{2}}\right\}\frac{1}{dist\left(x_{i},x_{j}\right)}, \end{array}$$

where *x*_*i*_ and *x*_*j*_ are the pixel intensity values of the biometric points and information verification parts of the face image respectively.

Carry out highlight detection and information fusion of multipose face image, select appropriate feature registration function to describe the feature points of multipose face image at different scales, and get the expression of face feature distribution as follows (11):

(11) $$\begin{array}{c} \begin{array}{c} F=\tilde{p}\left(x,y\right),\\ =p\left(x,y\right){\left(\frac{v\left(x\right)}{v\left(y\right)}\right)}^{1/2}, \end{array} \end{array}$$

where

(12) $$\begin{array}{c} \left\{\begin{array}{c} p\left(x,y\right)=\frac{k\left(x,y\right)}{v\left(x\right)},\\ v\left(x\right)=\underset{y}{\sum }\;k\left(x,y\right). \end{array}\right) \end{array}$$

The spatial neighborhood information is integrated into the amplitude detection of multipose face images, and the image segmentation algorithm is used for template matching of face images. According to the target matching results, the artificial neural network learning algorithm is used for image recognition.

#### 3.2.2. Face Image Recognition Output of Artificial Neural Network Learning

In fact, neural networks can be divided into biological and artificial ones. This paper mainly describes artificial neural networks. An artificial neural network (ANN) is a data model for information processing, which is similar to the synaptic connections of the brain.

The main component of the neural network is neurons. Its structure is shown in Figure 2. The input of each neuron requires the previous neuron to output data. The logic is clear and the structure is complete.

Usually, it is also called the logistic regression model. The structure of the neural network model is mainly in the hierarchical structure, which is composed of multiple neurons. As shown in Figure 3 below, this structure can display a neural network with hidden layers.

As shown in Figure 3*X*_1_, *X*_2_, and *X*_3_ are inputs of neural network. “+1” is the intercept term, also known as offset node. This neural network model contains three input units, three hidden units, and one output unit, and there is only one output node. The left is the input layer, the right is the output layer, and the middle layer is the hidden layer, which is fully connected with the input layer and the output layer. The values of all the nodes of the hidden layer cannot be displayed in the training sample.

RETRACTED

In different scales, appropriate feature registration functions are selected to describe the feature points of multipose face images, and the target pixel parallax analysis and key feature detection of multipose face images are carried out. According to the feature extraction results, the artificial neural network is used for face classification [15]. The artificial neural network is a three-layer network structure, and the input-output iteration equation of the artificial neural network classifier is as follows:

(13) $$\begin{array}{c} W\left(n+1\right)=W\left(n\right)-\eta \frac{\partial E}{\partial W}+\partial \Delta W\left(n\right), \end{array}$$

Assuming that the learning step of face recognition using an artificial neural network is *η*, after *n* steps of training and learning, the structural similarity feature decomposition algorithm is adopted to obtain the weighting coefficient of the face feature classifier as follows:

(14) $$\begin{array}{c} w_{sij}\left(n_{0}+1\right)=w_{sij}\left(n_{0}\right)-\eta_{sij}\frac{\partial J}{\partial w_{sij}}\text{.} \end{array}$$

Extract the facial image pose distribution information feature quantity, and use the artificial neural network classifier for feature calibration. The output detection statistics are as follows:

(15) $$\begin{array}{c} x\left(n\right)+\overset{p}{\underset{k=1}{\sum }}a_{i}x\left(n-k\right)=\overset{m}{\underset{r=0}{\sum }}b_{r}u\left(n-r\right)\text{.} \end{array}$$

In order to improve the accuracy of face feature classification by the artificial neural network, the adaptive learning coefficient *X*(*x*_1_, *x*_2_,…, *x*_*n*_) is introduced into the hidden layer of the neural network to extract the hidden features of occluded faces. According to the difference in biological features, the recognition result of the multipose face image is as follows:

(16) $$\begin{array}{c} x_{k+1}=x_{k}-A_{k}^{-1}g_{k}\text{.} \end{array}$$

Input the test sample *y* and training sample set *D* in the face database to be recognized to obtain the face feature distribution set *α*^(1)^ = [1/*l*, 1/*l*, ⋯,1/*l*]^T^, where is the number of face information in the training set [16, 17]. The artificial neural network classifier is constructed, and the weighted value of the neural network classifier is obtained as follows:

(17) $$\begin{array}{c} W_{ii}^{\left(t\right)}=\omega_{\theta }\left(e_{i}^{\left(t\right)}\right)=\frac{1}{1+\exp\;\left[\mu {\left(e_{i}^{\left(t\right)}\right)}^{2}-\mu \delta \right]}\text{.} \end{array}$$

Affine transformation is used for face feature separation, which is expressed as: $\hat{\alpha }={\left(D^{T}W^{\left(t\right)}D+\lambda \cdot I\right)}^{-1}D^{T}W^{\left(t\right)}y$, where *W*^(*t*)^ is the binary fitting result, *W*_*ii*_^(*t*)^=*ω*_*θ*_(*e*_*i*_^(*t*)^). Carry out a gray-scale sampling of multipose face features within the range of [0, 1], make ∑_*i*=1_^*n*^*ρ*_*θ*_(*e*^(*t*)^) < ∑_*i*=1_^*n*^*ρ*_*θ*_(*e*^(*t* − 1)^), and obtain the recognition output result: *y*_*rec*_^(*t*)^=*Dα*^(*t*)^. Let *t*=*t*+1, and then perform a global convergence analysis. When the quantity condition is met, the iteration is ended to realize face image recognition [18].

RETRACTED

## 4. Result Analysis

### 4.1. Simulation Experiment Analysis

The application performance of the proposed method in feature extraction of multipose face images is simulated [19]. The experiment is designed with MATLAB. The frame frequency of dynamic face image acquisition is 1200 kHz, the number of collected samples of the multipose face image is 2000, the training sample set is 200, the noise coefficient $\hat{m}$ = 0.24, the number of multipose face image blocks is 120, and the structural similarity is 0.12. The performance test index adopts the peak signal-to-noise ratio, which is defined as the following formula:

(18) $$\begin{array}{c} PSNR=20lg\;\frac{255}{MSE}=10\;dB, \end{array}$$

where $MSE=\sqrt{1/\left(M\times N\right)\underset{i}{\sum }\;{\left(f_{i}-{\hat{f}}_{i}\right)}^{2}}$ represents the normalized root mean square error and *f*, $\hat{f}$, respectively, represent the original image and the face image output after feature extraction, and the neighborhood window is taken as 9 x 9 [20].

According to the above simulation environment and parameter settings, the feature extraction results of face image recognition are obtained. It is known that the proposed method can effectively realize the recognition of multipose face images [21]. The performance comparison of face recognition is shown in Figure 4, and the comparison of recognition accuracy and time cost is shown in Figures 5 and 6.

By analyzing Figures 4, 5, and 6, it is known that the output signal-to-noise ratio of the method in this paper for multipose face image recognition is high, which indicates that the accuracy of face recognition is high, and the accurate recognition probability is better than the traditional method [22–25].

RETRACTED

## 5. Conclusion

To improve the ability to automatically recognize facial expressions, a variety of facial recognition function records are used to exclude facial features and facial recognition actions. This article introduces a multidimensional image recognition algorithm based on neural network education. The surrounding spatial data were aggregated to visually detect multiple facial images, and the angular properties of multiple facial images were obtained. Multiface image structured data is compared and compared to a random field RGB three-dimensional flat-moving Earth and multiface images are detected and aggregated. Appropriate registration functions were selected to explain the details of multiple facial images at different scales, which demonstrated the importance of parallax analysis of target pixels and the detection of multiple facial images. Image stabilization and automatic recognition are a combination of neural network learning and recording processes. The test results show that the higher the output compared to the noise, the higher the acceptable performance.

## Figures and Tables

**Figure 1:** Facial biological image information scanning recognition.

**Figure 2:** Neuron diagram.

**Figure 3:** Neural network.

**Figure 4:** Comparison of face recognition performance.

**Figure 5:** Comparison of accuracy under different iteration times.

**Figure 6:** Time cost comparison under different iteration times.

## Data Availability

The data used to support the findings of this study are available from the corresponding author upon request.
